# Hyper-osmolarity environment-induced oxidative stress injury promotes nucleus pulposus cell senescence *in vitro*

**DOI:** 10.1042/BSR20191711

**Published:** 2019-09-20

**Authors:** Jiawei Xu, Haopeng Li, Kai Yang, Shuai Guo, Jie Wang, Chaoshuai Feng, Huayou Chen

**Affiliations:** Department of Orthopedics, the Second Affiliated Hospital of Xi ’an Jiaotong University, Xi’an, 710004, Shaanxi, People’s Republic of China

**Keywords:** intervertebral disc, nucleus pulposus, osmolarity, oxidative stress, senescence

## Abstract

Nucleus pulposus (NP) cell senescence is involved in disc degeneration. The *in situ* osmolarity within the NP region is an important regulator of disc cell’s biology. However, its effects on NP cell senescence remain unclear. The present study was aimed to investigate the effects and mechanism of hyper-osmolarity on NP cell senescence. Rat NP cells were cultured in the *in situ*-osmolarity medium and hyper-osmolarity medium. The reactive oxygen species (ROS) scavenger N-acetylcysteine (NAC) was added along with the medium to investigate the role of oxidative injury. Cell cycle, cell proliferation, senescence associated β-galactosidase (SA-β-Gal) activity, telomerase activity, expression of senescence markers (p16 and p53) and matrix molecules (aggrecan and collagen II) were tested to assess NP cell senescence. Compared with the *in situ*-osmolarity culture, hyper-osmolarity culture significantly decreased cell proliferation and telomerase activity, increased SA-β-Gal activity and cell fraction in the G_0_/G_1_ phase, up-regulated expression of senescence markers (p16 and p53) and down-regulated expression of matrix molecules (aggrecan and collagen II), and increased intracellular ROS accumulation. However, addition of NAC partly reversed these effects of hyper-osmolarity culture on cellular senescence and decreased ROS content in NP cells. In conclusion, a hyper-osmolarity culture promotes NP cell senescence through inducing oxidative stress injury. The present study provides new knowledge on NP cell senescence and helps us to better understand the mechanism of disc degeneration.

## Introduction

Intervertebral disc (IVD) degenerative disease is common in orthopedic outpatients. It is a main contributor to disability that frustrates life quality of the patients, and brings a heavy medical cost to a family [1]. IVD is a cartilaginous tissue that consists of the central gelatinous nucleus pulposus (NP), the peripheral annulus fibrosus (AF) and the endplates [2]. Though the accurate pathogenesis of disc degeneration remains unknown until now, it is clear that the central NP region first exhibits degenerative changes during disc degeneration [3–5]. Therefore, lots of current biological therapies are aimed to restore the number and function NP cells.

The IVD is a connective structural between two adjacent vertebral bones. It plays an important role in transmitting and absorbing mechanical load to maintain the spine motion stability [6]. The disc NP tissue possesses a high hydrophily since it contains large amount of negatively charged proteoglycans [7]. Under the physiological conditions, IVDs experience various magnitudes and patterns of mechanical loads, which leads to the inflow and outflow of water through the NP tissue and the endplates, and ultimately changes the osmolarity within the disc NP tissue [8,9]. A previous study by Urban et al. [10] demonstrated that the *in situ* NP tissue osmolarity ranges between 450 and 550 mOsm/kg in a day. Theoretically, a higher magnitude of mechanical compression will cause a high osmolarity of NP tissue because more water will be extruded by it. Previously, increasing evidences have proved that a high magnitude often frustrates the healthy NP cell bioactivities [11–14]. Because the osmolarity changes are secondary changes of mechanical compression, we deduced that a high osmolarity within the NP region will be detrimental to the healthy NP biology.

Disc degeneration is a complex process that is characterized by age-related change or tissue destruction induced by multiple external stress [15]. Previously, lot of studies have identified the existence of senescent cells within the disc tissue [16–20]. These researches have reached a consensus that cell senescence increases with advancing of disc degeneration [18,19]. It has been established that oxidative stress is an important risk factor of disc cell senescence [21]. Previously, hyper-osmolarity is proved to activate oxidative stress and promote cell senescence or apoptosis in other cells [22–24]. However, the role and potential mechanism of hyper-osmolarity in regulating NP cell senescence are not well studied until now.

Therefore, the present study mainly aimed to investigate the effects of hyper-osmolarity on NP cell senescence, and whether the oxidative stress reaction is involved in this process. NP cell senescence was evaluated by senescence associated β-galactosidase (SA-β-Gal) activity, cell proliferation potency, telomerase activity, cell-cycle analysis, senescence marker’s expression (p16 and p53) and matrix homeostatic phenotype.

## Materials and methods

### Rat NP cell collection and culture

Thirty-three Sprague–Dawley rats were used in the present study. All animal experiments were finished at the Animal Experiment Center of the Second Affiliated Hospital of Xi ’an Jiaotong University. Rat NP cells were collected within 3 h after sacrifice as described by a previous study [12]. Briefly, after rat lumbar discs (L1–L6) were separated under the sterile conditions, the individual lumbar disc was harvested and then the central NP tissue was collected. Subsequently, NP tissue samples were digested by 0.02% collagenase (Sigma–Aldrich, U.S.A.) with continuous shaking. Finally, NP cell pellets were cultured in a standard DMEM/F12 medium supplemented with 10% fetal bovine serum (FBS, Gibco, U.S.A.) in a common humidified atmosphere (37°C, 21% O_2_ and 5% CO_2_). Then, the passage 2 NP cells were used in the next experiments. Specifically, NP cells were respectively cultured for 13 days in the medium with an *in situ* osmolarity (430 mOsm/kg) and a hyper-osmolarity (550 mOsm/kg). The value of *in situ*-osmolarity and hyper-osmolarity was designed according to the *in situ* NP tissue osmolarity (400–450 mOsm/kg) and the variation range of osmolarity in 1 day [10,25]. The sucrase was added into the DMEM/F12 medium to adjust osmolarity that was verified by a freezing point osmotic pressure instrument (SMC-30C, Tianjin Tianhe company, China). In addition, the reactive oxidative species (ROS) scavenger N-acetylcysteine (NAC, 5 mM, Beyotime, China) was added along with the culture medium of hyper-osmolarity group to investigate the role of oxidative stress in this process. The concentration of NAC was determined according to a previous study [11].

### Cell proliferation assay

Cell proliferation potency was evaluated by CCK-8 assay. Briefly, after NP cells seeded in six-well plate (4 × 10^3^ NP cells per well) were treated by medium with different osmolarities for 4 and 8 days, they were incubated with fresh DMEM/F12 medium supplemented with 10% (v/v) CCK-8 solution (Beyotime, China) for 30 min. Then, they were subjected to a multimode reader (Thermo, U.S.A.) to measure the absorbance value at a wavelength of 450 nm (OD 450). Finally, NP cell proliferation was reflected by the value of OD 450.

### SA-β-Gal staining assay

Briefly, after NP cells seeded in six-well plate were treated by medium with different osmolarities for 13 days, they were used to perform the SA-β-Gal staining assay according to the manufacturer’s instructions (Beyotime, China). Then, NP cells were observed under a light microscope (Olympus EX51, Japan). The ratio of staining-positive NP cells to the total NP cells was used to reflect NP cell senescence.

### Telomerase activity

Telomerase activity of NP cells was analyzed using a telomerase (TE) enzyme-linked immuno sorbent assay (ELISA) kit (Mlbio, China). Briefly, after NP cells seeded in six-well plate were treated by medium with different osmolarities for 13 days, they were lysed using RIPA lysis buffer (Beyotime, China). Then, the protein supernatant was used to analysis telomerase activity according to the manufacturer’s instructions. The standard substance in the test kit was used to create a standard curve. Telomerase activity (IU/l) of NP cells in each group was calculated based on the absorbance values at 450 nm and the standard curve.

### Cell-cycle analysis

NP cell cycle was analyzed by propidium iodide (PI, Beyotime, China) staining method. Briefly, after NP cells were treated by medium with different osmolarities for 13 days, they were dismissed by digestion with 0.25% trypsin without ethylene diamine tetraacetic acid (EDTA) and fixed by the cold ethanol for 24 h. Then, they were incubated with 50 μg/ml PI staining solution for 30 min at room temperature. Finally, the processed NP cells were subjected to a flow cytometry machine to analyze cell fraction in each cell-cycle phase (G_0_/G_1_, G_2_/M, S).

### ROS content

The ROS content within the NP cells was measured using a ROS detection kit (Beyotime, China). Briefly, after NP cells were treated by medium with different osmolarities for 13 days, 5 × 10^5^ NP cells in each group were stained with DCFH-CA (10 μM) for 20 min at 37°C. Finally, they were subjected to an automatic microplate reader (Thermo Fisher Scientific, U.S.A.) to measure the relative fluorescence units (RFU) at an excitation/emission wavelength of 490/585 nm. The RFU was used to reflect intracellular ROS content.

### Real-time PCR analysis

Total RNA was extracted from NP cells cultured in different osmolarity medium for 13 days using TRIzol reagent (Invitrogen, U.S.A.). Then, 1 μg of total RNA was reverse-transcribed into cDNA using a Reverse Transcription Kit (TIANGEN, China). Then, mRNA expression of target genes was detected using the S1000™ PCR instrument (Bio-Rad, U.S.A.). The SYBR Green Mix (DONGSHENG BIOTECH, China) was used to real-time detect amplification (50 ng cDNA template, 40 cycles: 20 s at 95°C, 30 s at 57°C, 30 s at 72°C). The primers of target genes were shown in the Table 1. β-actin was used as the internal gene. The mRNA expression of target genes was calculated with the method of 2^―ΔΔ*C*^_t_.

**Table 1:** Primers of target genes

Gene	Forward (5’–3’)	Reverse (5’–3’)
*β-actin*	CCGCGAGTACAACCTTCTTG	TGACCCATACCCACCATCAC
*Aggrecan*	ATGGCATTGAGGACAGCGAA	GCTCGGTCAAAGTCCAGTGT
*Collagen II*	GCCAGGATGCCCGAAAATTAG	CCAGCCTTCTCGTCAAATCCT
*P53*	CCTTAAGATCCGTGGGCGT	GCTAGCAGTTTGGGCTTTCC
*P16*	TACCCCGATACAGGTGATGA	TACCGCAAATACCGCACGA

### Western blot analysis

Expression of target molecules was analyzed by Western blot assay. Briefly, after total protein was extracted from NP cells treated by medium with different osmolarities for 13 days using the RIPA lysis buffer (Beyotime, China), they were subjected to SDS/PAGE and transferred to the PVDF membrane. Subsequently, the PVDF membranes were incubated with primary antibodies (β-actin: Cell Signaling Technology, #3700; p53: Cell Signaling Technology, #2524; p16: Novus, NBP2-37740) and horse radish peroxidase (HRP)-conjugated secondary antibodies (Beyotime, China). After protein bands were visualized using ECL Plus (Thermo, U.S.A.), their gray value were measured by the Quantity One software (Bio-Rad, U.S.A.). All protein expression of target molecules was normalized to β-actin.

### Statistical analysis

All data are presented as the mean ± standard error of the mean for three independent experiments (*n*=3). Each experiment was performed in triplicate. The statistical difference between groups was determined by one way analysis of variance (ANOVA) using SPSS 17.0 software. A probability value of <0.05 was regarded as significant.

## Results

### Cell proliferation of NP cells

After treatment by medium with different osmolarities for 4 and 8 days, NP cell proliferation was evaluated by CCK-8 assay. Results showed that hyper-osmolarity significantly suppressed NP cell proliferation on days 3 and 7 compared with the *in situ* osmolarity. However, addition of NAC partly increased NP cell proliferation in the hyper-osmolarity culture (Figure 1).

**Figure 1:** NP cell proliferation evaluated by CCK-8 assay Data are expressed as mean ± SD (*n*=3). *: Means a statistical difference (*P*<0.05) between two groups.

### SA-β-Gal activity of NP cells

SA-β-Gal activity is an important marker to reflect cellular senescence [16]. Our results showed that SA-β-Gal activity in the hyper-osmolarity culture significantly increased compared with that in the *in situ*-osmolarity culture. When the NAC was added along with the hyper-osmolarity culture medium, SA-β-Gal activity was partly inhibited (Figure 2).

**Figure 2:** SA-β-Gal activity of NP cells Magnification: 200×; scale = 100 μM; *n*=3. Data are expressed as mean ± SD. *: Means a statistical difference (*P*<0.05) between two groups.

### Telomerase activity of NP cells

Because telomerase is helpful to lengthen telomere during DNA duplicate, its activity is an important parameter to evaluate cellular senescence [26]. Results showed that hyper-osmolarity culture significantly decreased telomerase activity compared with the *in situ*-osmolarity culture, whereas the NAC partly increased telomerase activity of NP cells in the hyper-osmolarity culture (Figure 3).

**Figure 3:** Telomerase activity of NP cells Data are expressed as mean ± SD (*n*=3). *: Means a statistical difference (*P*<0.05) between two groups.

### NP cell cycle

Cell-cycle arrest is another indicator of cell senescence [27]. Results showed that NP cells in the hyper-osmolarity culture presented an increased cell fraction in G_0_/G_1_ phase and a decreased cell fraction in G_2_/M phase compared with the *in situ*-osmolarity culture. However, NAC partly reversed this result in the hyper-osmolarity culture (Figure 4).

**Figure 4:** Cell-cycle analysis of NP cells The cell fraction proportion of each cell cycle (G_0_/G_1_, S and G_2_/M) were calculated.

### ROS generation of NP cells

The oxidative stress induced by the accumulation of the intracellular ROS is involved in cellular senescence of disc cells [28,29]. Our results showed that ROS content in NP cells in the hyper-osmolarity culture is much higher than that in NP cells in the *in situ*-osmolarity culture, but it is expected to decrease after addition of NAC in the hyper-osmolarity culture (Figure 5).

**Figure 5:** Measurement of the intracellular reactive oxygen species (ROS) in NP cells Data are expressed as mean ± SD (*n*=3). *: Means a statistical difference (*P*<0.05) between two groups.

### Expression of matrix molecules in NP cells

Senescent cells often exhibit senescent-associated secretory phenotypes (SASP) which directly inhibits matrix anabolism [15]. To evaluate matrix homeostatic profile, expression of macromolecules (aggrecan and collagen II) of NP matrix was analyzed at both gene (Figure 6A) and protein (Figure 6B) levels. Results showed that their expression was down-regulated in the hyper-osmolarity culture compared with that in the *in situ*-osmolarity culture at both mRNA and protein levels, whereas this results was partly reversed by the addition of NAC into the medium of hyper-osmolarity culture.

**Figure 6:** Expression of matrix molecules (aggrecan and collagen II) in NP cells (**A**) Real-time PCR analysis. (**B**) Western blot analysis. Data are expressed as mean ± SD (*n*=3). *: Means a statistical difference (*P*<0.05) between two groups.

### Expression of senescence molecules in NP cells

Because cell senescence is often regulated by two classical ways: the replicative senescence (RS) regulated by the p53-p21-RB pathway and the stress-induced premature senescence (SIPS) regulated by the p16-RB pathway [30], the p16 and p53 are regarded as two cellular senescence markers. Here, our results showed that expression of p16 and p53 in NP cells in the hyper-osmolarity culture was significantly up-regulated compared with that in the *in situ*-osmolarity culture at both gene and protein levels, whereas addition of the NAC party inhibited their expression at both gene and protein levels in the hyper-osmolarity culture (Figure 7).

**Figure 7:** Expression of senescence-related molecules (p16 and p53) in NP cells (**A**) Real-time PCR analysis. (**B**) Western blot analysis. Data are expressed as mean ± SD (*n*=3). *: Means a statistical difference (*P*<0.05) between two groups.

## Discussion

Disc degeneration is a main contributor to low back pain [1]. Currently, its pathogenesis remains unclear to scholars and the effective biological treatments for regenerating degenerative disc are not realized. The osmolarity changes induced by mechanical compression in daily life is an obvious physicochemical feature in the NP region [8,9]. Previous studies have indicated that hyper-osmolarity obviously affects disc NP cell biology *in vitro* [9,31–39]. In the present study, we demonstrated for the first time that hyper-osmolarity culture promoted NP cell senescence and the aggravated oxidative stress injury was involved in this process. The present study sheds a new light on the important role of hyper-osmolarity in regulating NP cell senescence and helps us to further understand the mechanism of NP cell senescence during disc degeneration.

In daily life, the IVD is subjected to various mechanical stimuli, which leads to diurnal changes in osmolarity within the NP region due to the load-caused water extrusion and re-imbibition [8,9]. Previously, several studies have demonstrated that many disc cell’s biologies are affected by osmolarity, including matrix molecules (aggrecan, collagen II and collagen I) expression and cell viability [9,31–39]. In the present study, we found that hyper-osmolarity significantly decreased cell proliferation and telomerase activity, increased SA-β-Gal activity and cell fraction in G_0_/G_1_ phase, up-regulated expression of senescence markers (p16 and p53) and down-regulated expression of matrix molecules (aggrecan and collagen II) compared with the *in situ*-osmolarity culture. These results suggest that hyper-osmolarity culture promoted NP cell senescence compared with the *in situ*-osmolarity culture. In line with us, a previous study has demonstrated that hyper-osmolarity induced by glucose promotes senescence of human glomerular mesangial cells [23]. Theoretically, oxidative stress injury has been proved to participate disc cell senescence [28,29]. In the present study, we found that the promoted NP cell senescence was coincide with the increased intracellular ROS accumulation in the hyper-osmolarity culture, whereas the ROS scavenger NAC partly attenuated NP cell senescence in the hyper-osmolarity culture. This indicates that hyper-osmolarity can induce oxidative injury and thus cause disc NP cell senescence. Similarly, a study by Li et al. [22] has demonstrated that hyper-osmolarity induces cell apoptosis via initiating oxidative stress in primary human corneal epithelial cells.

However, the present study has several limitations. First, this is an *in vitro* study. Because adjusting the osmolarity value within the NP region *in vivo* is difficult to realize currently, we just investigate the effects of a hyper-osmolarity on NP cell senescence in a cell culture system. Second, no specific cellular markers have been found to distinguish NP cells from notochordal cells. The isolated cells may contain both NP cells and notochordal cells since the existence of notochordal cells within the rat disc NP tissue.

In conclusion, we investigated the effects and mechanism of hyper-osmolarity on NP cell senescence. Our results demonstrated that hyper-osmolarity accelerated NP cell senescence though inducing oxidative injury. The present study provides new knowledge on NP cell senescence and helps us to better understand mechanism of disc degeneration.

## Abbreviations

CCK-8: cell counting kit-8
IVD: intervertebral disc
NAC: N-acetylcysteine
NP: nucleus pulposus
OD: optical density
PI: propidium iodide
RFU: relative fluorescence unit
RIPAr: radio-immunoprecipitation assay
ROS: reactive oxidative species
SA-β-Gal: senescence associated β-galactosidase
